The article "Proxalutamide Reduces the Rate of Hospitalization for COVID-19 Male Outpatients: A Randomized Double-Blinded Placebo-Controlled Trial" was retracted in 2022. Reasons: errors in the methods; unreliable results or conclusions; concerns about the data.

# Proxalutamide Reduces the Rate of Hospitalization for COVID-19 Male Outpatients: A Randomized Double-Blinded Placebo-Controlled Trial

**DOI:** 10.3389/fmed.2021.668698

**Published:** 2021-07-19

**Authors:** John McCoy, Andy Goren, Flávio Adsuara Cadegiani, Sergio Vaño-Galván, Maja Kovacevic, Mirna Situm, Jerry Shapiro, Rodney Sinclair, Antonella Tosti, Andrija Stanimirovic, Daniel Fonseca, Edinete Dorner, Dirce Costa Onety, Ricardo Ariel Zimerman, Carlos Gustavo Wambier

**Affiliations:** ^1^Applied Biology, Inc. Irvine, CA, United States; ^2^Department of Endocrinology, Corpometria Institute, Brasilia, Brazil; ^3^Dermatology Department, Ramón y Cajal Hospital, Madrid, Spain; ^4^Department of Dermatology and Venereology, University Hospital Center “Sestre Milosrdnice”, Zagreb, Croatia; ^5^Ronald O. Perelman Department of Dermatology, New York University School of Medicine, New York, NY, United States; ^6^Sinclair Dermatology, Melbourne, VIC, Australia; ^7^Department of Dermatology and Cutaneous Surgery, Miller School of Medicine, University of Miami, Miami, FL, United States; ^8^School of Medicine, European University Cyprus, Nicosia, Cyprus; ^9^Intensive Care Unit, Samel Hospital, Manaus, Brazil; ^10^Hospital da Brigada Militar, Porto Alegre, Brazil; ^11^Department of Dermatology, Alpert Medical School of Brown University, Providence, RI, United States

**Keywords:** proxalutamide, COVID-19, androgen receptor, antiandrogens, androgenetic alopecia, anti-androgen therapy, transmembrane protease serine 2, TMPRSS2

## Abstract

Antiandrogens have demonstrated a protective effect for COVOD-19 patients in observational and interventional studies. The goal of this study was to determine if proxalutamide, an androgen receptor antagonist, could be an effective treatment for men with COVID-19 in an outpatient setting. A randomized, double-blinded, placebo-controlled clinical trial was conducted at two outpatient centers (Brasilia, Brazil). Patients were recruited from October 21 to December 24, 2020 (clinicaltrials.gov number, NCT04446429). Male patients with confirmed COVID-19 but not requiring hospitalization (COVID-19 8-point ordinal scale <3) were administered proxalutamide 200 mg/day or placebo for up to 7 days. The primary endpoint was hospitalization rate at 30 days post-randomization. A total of 268 men were randomized in a 1:1 ratio. 134 patients receiving proxalutamide and 134 receiving placebo were included in the intention-to-treat analysis. The 30-day hospitalization rate was 2.2% in men taking proxalutamide compared to 26% in placebo, *P* < 0.001. The 30-day hospitalization risk ratio was 0.09; 95% confidence interval (CI) 0.03–0.27. Patients in the proxalutamide arm more frequently reported gastrointestinal adverse events, however, no patient discontinued treatment. In placebo group, 6 patients were lost during follow-up, and 2 patients died from acute respiratory distress syndrome. Here we demonstrate the hospitalization rate in proxalutamide treated men was reduced by 91% compared to usual care.

The article "Proxalutamide Reduces the Rate of Hospitalization for COVID-19 Male Outpatients: A Randomized Double-Blinded Placebo-Controlled Trial" was retracted in 2022. Reasons: errors in the methods; unreliable results or conclusions; concerns about the data.

## Introduction

Androgen signaling plays a central role in SARS-CoV-2 infectivity. SARS-CoV-2 cell entry is mediated by priming of viral spike proteins by the androgen-promoted enzyme, transmembrane protease, serine 2 (TMPRSS2). Structural modification of viral spike proteins enhances binding of SARS-CoV-2 to angiotensin converting enzyme 2 (ACE2) and facilitates viral entry into cells. Thus, targeting the transcription of TMPRSS2 with antiandrogens can affect viral cell entry (1, 2). It has been demonstrated that ACE2 and TMPRSS2 levels in lung and cardiac cells are reduced by antiandrogens (3, 4). Conversely, patients with androgen sensitive phenotypes have been shown to have increased COVID-19 disease burden. The androgen-mediated phenotype androgenetic alopecia (AGA) has been associated with greater COVID-19 disease severity (5–7). Further, the progression of AGA in hospitalized men showed a direct association with COVID-19 disease severity; men with more advanced AGA were more likely to require intensive care or die (5, 8).

In a large population based study of COVID-19 patients in northern Italy, it was reported that prostate cancer patients undergoing androgen depravation therapy (ADT) had lower SARS-CoV-2 infection rates compared to prostate cancer patients not receiving ADT (OR 4.05; 95% CI 1.55–10.59) (9). Similarly, we have reported the protective effect of 5-alpha-reductase inhibitors (5ARi) for men with COVID-19 in two observational studies (10, 11). 5ARis such as finasteride and dutasteride block the conversion of testosterone to a more potent intracellular androgen, dihydrotestosterone (4). In a study of 77 men hospitalized with COVID-19 we found that among chronic antiandrogen users (primarily dutasteride) 8% were admitted to the ICU, compared to 58% of men not taking antiandrogens (*p* = 0.0015) (10). Moreover, the frequency of COVID-19 symptoms among men with AGA was drastically reduced in users of 5ARis in an outpatient setting. A statistically significant reduction in the frequency of 20 of 29 clinical symptoms was observed in 5ARi users compared to non-users. For example, 38 and 2% of men presented with low-grade fever, 60 and 6% with dry cough, and 88% and 15% reported anosmia in the non-5ARi and 5ARi groups, respectively (11). In a randomized, placebo-controlled trial, early antiandrogen therapy with dutasteride resulted in faster recovery from symptoms, improvement in inflammatory markers, and reduced detection rates of SARS-CoV-2 in nasopharyngeal swabs after 7 days compared to placebo (35.7 vs. 88.2%, *p* = 0.0094) (12). Similarly, in a randomized clinical trial that enrolled 80 hospitalized men, the use of finasteride (a 5ARi with a shorter half-life than dutasteride) was associated with improvement in oxygen saturation by day 5, and a 75% lower mortality rate (13).

The article "Proxalutamide Reduces the Rate of Hospitalization for COVID-19 Male Outpatients: A Randomized Double-Blinded Placebo-Controlled Trial" was retracted in 2022. Reasons: errors in the methods; unreliable results or conclusions; concerns about the data.

Proxalutamide is a potent second-generation non-steroidal androgen receptor (AR) antagonist (14). AR antagonists competitively inhibit androgen hormones from binding to the AR, which prevents AR dimerization and binding of AR dimers to DNA (15). We have previously reported our preliminary analysis of the effects of proxalutamide 200 mg per day in COVID-19 patients, which showed an overall 74% reduction in nasopharyngeal detection of SARS-CoV-2 on the 7th day of treatment (16). The objective of this study was to evaluate the efficacy of proxalutamide in preventing hospitalization in males diagnosed with COVID-19 in an outpatient setting.

## Methods

### Study Design and Oversight

This was double-blinded, randomized, placebo-controlled clinical trial of proxalutamide for the treatment of male outpatients with COVID-19 (NCT04446429). The study was approved by the Brazilian National Ethics Committee: #4.282.108; process number (CAAE) 36703320.8.0000.0023 of the Comitê de Ética em Pesquisa (CEP), Comitê Nacional de Ética em Pesquisa (CONEP), Ministry of Health [Ministério da Saúde (MS)] (CEP/CONEP/MS). All patients were volunteers and received no financial compensation. All patients gave informed consent.

### Study Population and Covariates

Patients were recruited through social media or by referral from primary care physicians from October 21 to December 24, 2020. Potential study patients presented one of two outpatient centers (Centro Clínico Advance or Exame Imagem e Laboratorio, Brasilia, Brazil) for suspected COVID-19. Self-referred patients that contacted the study sites for participation underwent a medical screening visit prior to randomization. Nasopharyngeal swabs were collected from all potential patients by trained medical personal. SARS-CoV-2 status was confirmed by real-time reverse transcription polymerase reaction (rtPCR) testing following the Cobas rtPCR kit protocol (Automatized Platform, Roche, USA).

The inclusion criteria were: males with mild COVID-19 disease (COVID-19 8-point ordinal scale <3), positive rtPCR for SARS-CoV2 within 7 days of randomization, initiation of symptoms 7 days prior to randomization, creatinine below 1.5 times the upper limit of normality (ULN), alanine transferase (ALT) below 3.0 times the ULN, total bilirubin below 2.0 times the ULN, and International Normalized Ratio of Prothrombin Time below 1.5 times the ULN, and age 18 years or older. The exclusion criteria were: signs of severe COVID-19 including respiratory rate >30 breaths/min, tachycardia >120 beats per minute, systolic and diastolic arterial blood pressure <90 and <60 mmHg, respectively, criteria for hospitalization at the time of randomization, uncontrolled types 1 or 2 diabetes mellitus or hypertension, congestive heart failure (CHF) grades 3 or 4 (New York Heart Association), left ventricle ejection rate below 50%, rate corrected Q-T interval above 450 mm in the electrocardiogram, HIV, active hepatitis B or C, active syphilis, cancer diagnosed in the past 5 years (except for skin and thyroid cancer), and refusal to use condom in the 90 days following treatment.

The article "Proxalutamide Reduces the Rate of Hospitalization for COVID-19 Male Outpatients: A Randomized Double-Blinded Placebo-Controlled Trial" was retracted in 2022. Reasons: errors in the methods; unreliable results or conclusions; concerns about the data.

Baseline characteristics, comorbidities, test results, and medications used were recorded. For each patient, the age, frequency and duration of medication used and the following pre-existing conditions were recorded: type 2 diabetes, hypertension, obesity (defined as body mass index >30 kg/cm^2^), and chronic obstructive pulmonary disease. The pre-existing conditions recorded were chosen based on previous drug trials in COVID-19.

### Procedures

Patients were randomized to receive either proxalutamide 200 mg/day for up to 7 days or placebo. Proxalutamide 200 mg and placebo were manufactured to appear identical (Kintor Pharmaceuticals Ltd., Suzhou, China). A blocked randomization list was created with block size of 10 and the sequence of dispensing was followed throughout the trial. The group assignment was known only to the study monitor. The patients and doctors directly managing patient care were blinded to the study group allocation until the close of the study. Patients were instructed to take one tablet once a day. The telephone contact and clinical follow-up were independently performed by study assistants that were blinded to group assignments. No changes in the randomization process occurred during the trial.

Previous prescriptions from referring medical doctors, initiated upon the diagnosis of COVID-19, were continued. All new patients, i.e., those not under ongoing care of a primary physician, were offered the usual care medications defined in the study protocol. Usual care consisted of various combinations of medications and was individualized to each patient's needs. Azithromycin 500 mg per day for 5 days and nitazoxanide 500 mg twice a day for 6 days were offered to all new study patients. The following medications were prescribed as needed: dipyrone, paracetamol, ondansetron, dexamethasone, rivaroxaban, and enoxaparin. In cases of hospitalization, additional drugs were prescribed according to the clinical judgement of the hospital staff. Treatment compliance with study drugs was not monitored during the trial. Usual care medications prescribed by doctors outside of the trial were not documented.

The article "Proxalutamide Reduces the Rate of Hospitalization for COVID-19 Male Outpatients: A Randomized Double-Blinded Placebo-Controlled Trial" was retracted in 2022. Reasons: errors in the methods; unreliable results or conclusions; concerns about the data.

### Protocol Modifications

The initial protocol approved by the IRB proposed the use proxalutamide 200 mg per day for 3 days only (approval #4.282.108). However, after the first safety analysis conducted from Oct 30 to Nov 01 (35 patients randomized), the safety committee observed that 3 patients allocated in the same group experienced unexpected relapse of COVID-19 symptoms after a few days of interruption of the investigational product. The study director agreed to unblind the 3 patients, which were observed to be from the proxalutamide group. The protocol was amended to change the posology from one tablet per day for 3 days to 1 tablet per day for 7 days (IRB approval #4.513.428). Upon study closing, a total of 75 patients were randomized and given bottles with 3 tablets (38 received proxalutamide), and a total of 193 patients were randomized and given bottles with 7 tablets (96 received proxalutamide).

### Study Outcomes

The primary outcome for the study was the percentage of patients hospitalized due to COVID-19. The COVID-19 8-point ordinal scale was used for screening as well as identifying patients as hospitalized. The 8-point ordinal scale is defined as: 8. Death; 7. Hospitalized, on invasive mechanical ventilation or extracorporeal membrane oxygenation (ECMO); 6. Hospitalized, on non-invasive ventilation or high flow oxygen devices; 5. Hospitalized, requiring supplemental oxygen; 4. Hospitalized, not requiring supplemental oxygen- requiring ongoing medical care (COVID-19 related or otherwise); 3. Hospitalized, not requiring supplemental oxygen—-no longer requires ongoing medical care; 2. Not hospitalized, limitation on activities; 1. Not hospitalized, no limitations on activities. Subjects were considered hospitalized if they achieved score >3 at any time during the 30 days post randomization.

### Statistical Analysis

Sample size estimate was based on a report by Riccardo et al. (17). In the report it was shown that in Italy the hospitalization rate was as high as 20% among adults above the age of 65 tested positive for SARS-CoV-2. Further, Montopoli et al. (9) reported that males represent 60% of hospitalized patients; therefore, we estimated that the 30-days rate of hospitalization of males over the age of 65, testing positive for SARS-CoV-2 would be ~30%. For the assumed efficacy of proxalutamide as a treatment for COVID-19, we estimated a 50% reduction in the hospitalization rate. Two hundred thirty-six patients are required to have 80% chance of detecting, as significant at the 5% level, a reduction in hospitalization rate from 30% in the control group to 15% in the proxalutamide group. Adjusting for non-compliance/cross-over of 2.5% in each group, we estimated a total of 262 patients (131 in each arm).

The article "Proxalutamide Reduces the Rate of Hospitalization for COVID-19 Male Outpatients: A Randomized Double-Blinded Placebo-Controlled Trial" was retracted in 2022. Reasons: errors in the methods; unreliable results or conclusions; concerns about the data.

Hospitalization risk ratio was used as the measure of efficacy in the analysis of the primary outcome. Kaplan-Meier estimates were used to evaluate the differences of hospitalization rates throughout the 30-days post-randomization observation period. Under the intention-to-treat analysis, all patients that were randomized and had ongoing consent to be evaluated for outcomes were included. Chi-squared test for independent proportions was adopted with statistical significance was set at *P* < 0.05. Stata/SE 17.0 for Mac (StataCorp, TX, USA) was used to perform all statistical analysis.

## Results

Two hundred sixty-eight men were randomized to the study. One hundred thirty-four men were randomized to the proxalutamide arm and 134 men were assigned to placebo. Six patients in the placebo arm discontinued treatment and withdrew consent. A total of 134 patients from the proxalutamide group and 128 patients from the placebo group were followed throughout the study period. The six patients from the placebo arm that were not followed were assumed to be non-hospitalized (COVID-19 8-point ordinal scale 1) and were included in the intention-to-treat analysis. The flow chart of patients recruited into the study is shown in Figure 1. Baseline characteristics of the two study groups are displayed in Table 1. Concomitant treatments were difficult to assess owing to the outpatient nature of the sampled population and were not monitored.

**Figure 1:** Enrollment and analyzed population.

**Table 1:** Baseline characteristics of the study arms.

**Characteristics**	**Overall** ***N* = 268**	**Proxalutamide** ***N* = 134**	**Placebo** ***N* = 134**
Age (years), median (IQR)	45 (17)	45 (19)	46 (15)
**Coexisting conditions, no. (%)**			
Type 2 diabetes	21 (8)	11 (8)	10 (7)
Hypertension	55 (21)	33 (25)	22 (16)
Chronic obstructive pulmonary disease	1 (0)	1 (0)	0 (0)
BMI > 30 kg/m^2^	43 (16)	22 (16)	21 (16)
**No. of coexisting conditions, no. (%)**			
0	158 (59)	74 (55)	84 (63)
1	49 (18)	29 (22)	20 (15)
2+	55 (21)	31 (23)	24 (18)
**Baseline 8-point ordinal scale score**			
1	160 (60)	63 (47)	97 (72)
2	108 (40)	71 (53)	37 (28)

During the 30-day post-randomization period, 3 patients (2.2%) in the proxalutamide group vs. 35 (26.1%) in the placebo group were hospitalized (Table 2). The 30-day hospitalization risk ratio was 0.09 [95% confidence interval (CI), 0.03–0.27], i.e., the hospitalization rate in proxalutamide treated men was reduced by 91% compared to placebo. The risk difference was −0.24 (95% CI, −0.32 to −0.16).

The article "Proxalutamide Reduces the Rate of Hospitalization for COVID-19 Male Outpatients: A Randomized Double-Blinded Placebo-Controlled Trial" was retracted in 2022. Reasons: errors in the methods; unreliable results or conclusions; concerns about the data.

**Table 2:** IQR, interquartile range; BMI, body mass index.

**Characteristic, no. (%)**	**Proxalutamide** ***N* = 134**	**Placebo** ***N* = 134**
Hospitalizations	3 (2)	35 (26)
Supplemental oxygen	2 (1)	33 (25)
Non-invasive ventilation	0 (0)	19 (14)
High flow oxygen devices	1 (1)	26 (19)
Invasive mechanical ventilation	0 (0)	17 (13)
Extracorporeal membrane oxygenation	0 (0)	6 (4)
Vasopressors	0 (0)	12 (9)
Death	0 (0)	2 (1)
**Day 15—8-point ordinal scale score, no. (%)**		
1	129 (96)	83 (62)
2	4 (3)	28 (21)
3	0 (0)	2 (1)
4	0 (0)	1 (1)
5	0 (0)	3 (2)
6	1 (1)	4 (3)
7	0 (0)	12 (9)
8	0 (0)	1 (1)
**Day 30—8-point ordinal scale score, no. (%)**		
1	132 (99)	104 (78)
2	2 (1)	17 (13)
3	0 (0)	0 (0)
4	0 (0)	4 (3)
5	0 (0)	4 (3)
6	0 (0)	0 (0)
7	0 (0)	3 (2)
8	0 (0)	2 (1)

A summary of the distribution of COVID-19 8-point ordinal scale scores at day 15 and day 30 post-randomization is included in Table 2. At day 30, 12 patients were still hospitalized in the placebo group, compared to zero in the proxalutamide arm. Figure 2 shows the cumulative hospitalization rates over the follow-up period of 30-days post-randomization. The 3 patients that were hospitalized in the proxalutamide group had later hospitalizations compared to the placebo group, which showed a higher rate of hospitalizations in the first 10 days. After 10 days, the rate of hospitalization was similar between groups.

**Figure 2:** Kaplan-Meier estimates of proportion admitted to hospitals due to COVID-19 during the 30-day post-randomization follow-up.

A summary of treatment emergent adverse events (TEAEs) is presented in Table 3. Gastrointestinal TEAEs were more frequent in the proxalutamide group: diarrhea (21% proxalutamide vs. 9% placebo), and nausea (14% proxalutamide vs. 6% placebo). Death within 30 days of enrollment in the study was reported for 2 patients (1.6%) in the placebo group. No deaths were reported in the proxalutamide group (Table 3). In the placebo arm, the primary cause of death was reported as acute respiratory distress syndrome (ARDS) resulting from progressive COVID-19 disease.

**Table 3:** Summary of treatment emergent adverse events (TEAEs).

**Characteristic**	**Proxalutamide** ***N* = 134**	**Placebo** ***N* = 128**	***P***
1 or more TEAE, no. (%)	82 (61.2%)	116 (90.6%)	
**General, no. (%)**			
Disease progression	4 (3)	43 (34)	<0.001
Hypoxemia (>4% decrease or reaching SpO_2_ <92%)	3 (2)	36 (28)	<0.001
Tachycardia	6 (4)	45 (35)	<0.001
Fatigue	1 (1)	71 (55)	<0.001
Shortness of breath	4 (3)	40 (31)	<0.001
Fever	2 (1)	34 (27)	<0.001
Dehydration	20 (15)	51 (39)	<0.001
Increase in ALT or AST (over the ULN)	4 (3)	22 (17)	<0.001
**Gastrointestinal, no. (%)**			
Diarrhea	39 (28)	20 (16)	0.009
Dyspepsia or heartburn	23 (17)	6 (5)	0.001
Abdominal pain or discomfort	22 (16)	18 (14)	0.596
Nausea	21 (16)	15 (12)	0.353
Vomiting	4 (3)	6 (5)	0.472
**Nervous system, no. (%)**			
Headache	1 (1)	12 (9)	0.001
Ageusia	13 (10)	23 (18)	0.052
Anosmia	14 (10)	26 (20)	0.026
Diffuse sweating	48 (36)	5 (4)	<0.001
Orthostatic dizziness	6 (4)	8 (6)	0.524
**Musculoskeletal, no. (%)**			
Arthralgia	5 (4)	22 (17)	<0.001
Muscle pain	3 (2)	39 (30)	<0.001
Lower back pain	11 (8)	24 (19)	0.012
Upper back pain	5 (4)	12 (9)	0.064
Pain in extremity	2 (1)	4 (3)	0.377
**Skin and subcutaneous tissue, no. (%)**			
Skin Lesions	10 (7)	7 (5)	0.512
Total TEAE, no.^*^	276	591	–

*Patients with multiple adverse events were counted more than once in the total TEAEs.

The article "Proxalutamide Reduces the Rate of Hospitalization for COVID-19 Male Outpatients: A Randomized Double-Blinded Placebo-Controlled Trial" was retracted in 2022. Reasons: errors in the methods; unreliable results or conclusions; concerns about the data.

*ALT, alanine aminotransferase; AST, aspartate aminotransferase; ULN, Upper Limit of Normality*.

## Discussion

These results show the improvement of clinical outcomes in men with COVID-19 after the use of proxalutamide 200 mg per day. We have previously reported the protective effect of the 5-alpha-reduactase inhibitor, dutasteride, in men with COVID-19, both in hospitalized patients and in an outpatient setting (10–12). As dutasteride has a half-life of 5 weeks and carries a labeled contraindication for the use in women of childbearing age (18, 19), we were keen to explore an antiandrogen that could be applied more broadly. Proxalutamide has been evaluated for 28 days in Phase 1 safety studies for both men and women; furthermore, the half-life is ~22 h (20). As such, proxalutamide would be more suitable for application in men and women. We are currently completing an outpatient trial focused on female patients (NCT04853134). Additionally, we have completed a randomized, placebo-controlled trial of proxalutamide for male and female hospitalized COVID-19 patients (NCT04728802). Future trials should also explore other non-steroidal antiandrogens (NSAA) with proven safety data in the treatment of COVID-19, e.g., apalutamide, enzalutamide, darolutamide, bicalutamide, or flutamide.

The dosage used in this trial, 200 mg for up to 7 days was effective in reducing the hospitalization rates by 91%. All patients that were hospitalized in the proxalutamide group took proxalutamide for 7 days and were hospitalized only after stopping the medication, which suggests a relapse of inflammation or viral activity. Although no patient was hospitalized with 3 days of proxalutamide, the initial number of patients was too low to draw conclusions. It is still unknown if different posology could improve efficacy in the outpatient setting. However, higher dosages, a higher initial loading dose, or a longer treatment course could be explored in future trials. For example, 300 mg per day for 14 days has been used in hospitalized patients (NCT04728802). Additionally, a loading dosage 600 mg followed by 200 mg per day for 7 days has been reported in a single case (21).

The article "Proxalutamide Reduces the Rate of Hospitalization for COVID-19 Male Outpatients: A Randomized Double-Blinded Placebo-Controlled Trial" was retracted in 2022. Reasons: errors in the methods; unreliable results or conclusions; concerns about the data.

SARS-CoV-2 cell entry into type II pneumocytes is blocked by TMPRSS2 inhibitors (22, 23) and TMPRSS2 transcription inhibitors (antiandrogens) (1, 3). We expect an antiandrogen-class effect on protection from COVID-19, which may be explained by mechanisms distinct from the androgen-mediated SARS-COV-2 cell entry mechanism (24). A non-immunosuppressive anti-inflammatory effect may occur, as the activation of the androgen receptor by dihydrotestosterone leads to increased IL-6 production in macrophages, delaying repair of injury (25). Furthermore, NSAA use was associated with a reduction in plasma IL-6 and TNF post-trauma (26), and reduction in inflammatory response induced by radiation (27). Of note, the androgen receptor may be activated though the IL-6 STAT3 activation pathway (3, 28). More research is needed to elucidate the mechanism of NSAA and other antiandrogens on COVID-19.

We acknowledge that there are important limitations in the present study. Primarily, no direct monitoring of treatment compliance was conducted; additionally, owing to the open recruitment, complete data for the usual care medications was not available to be analyzed. This has the potential to mask the effects of proxalutamide or to introduce imbalances in the application of usual care medication. However, in the usual care treatment, only nitazoxanide has been shown to have potential efficacy in placebo-controlled trials (29–31) and this drug was offered to all new patients. Further, the randomization of patients to each trial study arm would mitigate any uneven distribution of usual care medications, if they existed. Second, the protocol change from a 3-day to a 7-day intervention schedule could have masked differences between treatment with placebo and proxalutamide, i.e., treatment with 3 days of proxalutamide may have been ineffectual. Nevertheless, proxalutamide retained its efficacy in intention-to-treat analysis. Finally, the six patients that withdrew from the study were all from the placebo arm. To account for this, we assumed the greatest bias against the tested drug, and included all six patients as non-hospitalized in the intention-to-treat analysis.

The article "Proxalutamide Reduces the Rate of Hospitalization for COVID-19 Male Outpatients: A Randomized Double-Blinded Placebo-Controlled Trial" was retracted in 2022. Reasons: errors in the methods; unreliable results or conclusions; concerns about the data.

Here we demonstrate that proxalutamide was a benefit to men with mild to moderate COVID-19. Male outpatients with SARS-CoV-2 were 91% less likely to be hospitalized vs. those treated with placebo. We hope the results of this study encourage more trials of proxalutamide and other antiandrogens for the treatment of COVID-19.

## Conclusion

In COVID-19 male outpatients, treatment with proxalutamide reduced the rate of hospitalization by 91%. The results of the present study further elucidate the protective impact of early antiandrogen treatment for COVID-19 in the outpatient setting. Further studies of antiandrogen therapies in COVID-19 patients are needed.

## Data Availability Statement

The original contributions presented in the study are included in the article/supplementary material, further inquiries can be directed to the corresponding author/s.

## Ethics Statement

The studies involving human participants were reviewed and approved by an ethics committee, registered with clinicaltrials.gov (NCT04446429), and also approved by Brazilian National Ethics Committee [Approval number #4.282.108; CAAE:36703320.8.0000.0023; Comitê de Ética em Pesquisa (CEP) of the Comitê Nacional de Ética em Pesquisa (CONEP) of the Ministry of Health (MS)] (CEP/CONEP/MS). The patients/participants provided written informed consent to participate in this study.

## Author Contributions

JM, AG, CW, and FC contributed to conception and design of the study. FC, DF, ED, and DO collected clinical data. AG and JM analyzed and prepared data. JM and CW prepared first draft. All authors contributed to manuscript revision, read, and approved the submitted version.

## Conflict of Interest

Kintor Pharmaceuticals, Ltd. manufactures and plans to market proxalutamide, and has an investigational new drug (IND) application under United States Food and Drugs Administration to conduct a Phase 3 study for proxalutamide for COVID-19. Applied Biology, Inc. has patents pending regarding antiandrogen therapy for COVID-19. AG and JM are employees of Applied Biology, Inc. FC has served as a clinical director for Applied Biology, Inc. CW, JS, and RS has served as an advisor to Applied Biology, Inc. The remaining authors declare that the research was conducted in the absence of any commercial or financial relationships that could be construed as a potential conflict of interest.
